# Robust Adaptive Self-Structuring Neural Network Bounded Target Tracking Control of Underactuated Surface Vessels

**DOI:** 10.1155/2021/2010493

**Published:** 2021-12-21

**Authors:** Haitao Liu, Jianfei Lin, Guoyan Yu, Jianbin Yuan

**Affiliations:** ^1^School of Mechanical and Power Engineering, Guangdong Ocean University, Zhanjiang 524088, China; ^2^Southern Marine Science and Engineering Guangdong Laboratory (Zhanjiang), Zhanjiang 524000, China

## Abstract

This paper studies the target-tracking problem of underactuated surface vessels with model uncertainties and external unknown disturbances. A composite robust adaptive self-structuring neural-network-bounded controller is proposed to improve system performance and avoid input saturation. An extended state observer is proposed to estimate the uncertain nonlinear term, including the unknown velocity of the tracking target, when only the measurement values of the line-of-sight range and angle can be obtained. An adaptive self-structuring neural network is developed to approximate model uncertainties and external unknown disturbances, which can effectively optimize the structure of the neural network to reduce the computational burden by adjusting the number of neurons online. The input-to-state stability of the total closed-loop system is analyzed by the cascade stability theorem. The simulation results verify the effectiveness of the proposed method.

## 1. Introduction

In recent years, the tracking control problem of underactuated surface vessels (USVs) has attracted the attention of many researchers. The design of motion controllers for USVs is extremely important due to their applications in target search, resource exploration, oceanographic mapping, and ocean dynamic surveillance [1, 2]. The primary difficulty of USV tracking control is that it cannot satisfy various degrees of freedom to achieve independent power. Additionally, in the case of model uncertainties and unknown low-frequency time-varying external disturbances, the design of the USV nonlinear tracking controller is particularly difficult [3–5]. The challenges of controller design are as follows:

1. At present, general surface vessels can provide two degrees of freedom: control input surge and yaw. These vessels are underactuated systems in which the number of independent actuators (input) is less than the controlled degrees of freedom (output) [6–11].
2. It is difficult or impossible to design an accurate vessel model. For example, the Coriolis and centripetal terms and hydrodynamic damping forces in the model cannot be accurately determined [12–14].
3. The external unknown disturbances caused by waves, wind, and ocean currents seriously affect the stability and robustness of the USV control system [15].

Model uncertainties have a serious impact on the performance and stability of the control system. When external unknown disturbances are added, the robustness of the system worsens. Many model-based USV tracking control methods have been proposed. The tracking control method was based on the Lyapunov theorem and backstepping technique in [16]. In [17], the controller was designed through the nonlinear coordinate transformation of the vessel model to obtain global uniformity and final boundedness. To address the unknown nonlinear components caused by the uncertainty of the model parameters, the adaptive control method was proposed to solve the tracking control problem and improve the system's robustness [18, 19]. In [18], by updating the adaptive law, a parameter compression algorithm was developed to address the problems of model uncertainty and unknown disturbances in a more concise way. Fuzzy control combined with minimum learning parameters and a fuzzy adaptive control method with state feedback was proposed to address model uncertainties in [19]. Recently, in USV tracking control, a variety of NN adaptive technologies were designed to compensate for model uncertainties [20–25]. Under the conditions of uncertain model parameters and unknown nonlinearity, an adaptive observer based on NNs was developed to estimate USV speed with uncertain terms [20]. In [21], a robust controller based on the traditional RBFNN was proposed to compensate for the dynamic uncertainty. To ensure performance, an adaptive NN controller was developed to compensate for model uncertainties in [22, 23].

In motion control, target control has attracted more attention [26–28]. In [26], a measuring target velocity observer was developed to assist in tracking the upper target under the constraints of position, angle, and speed. In [27], the range and angle of the underwater robot relative to the tracking target were transformed into a dynamic second-order model with open-loop error. Multilayer NN and robust controller with adaptive parameters were used to achieve target-tracking control. In [28], based on the line-of-sight (LOS) measurements of angle and range, a target-tracking controller was proposed. Fuzzy control [29, 30] has been validated in various practical applications such as the control of USVs. In [31], an adaptive output-feedback fuzzy control was proposed by using a fuzzy logic system (FLS) to approximate the model uncertainties. In particular, during the target-tracking process, only the target's instantaneous movement information is available. The above trajectory control strategy can obtain the required tracking information, including position and velocity, but without considering the unknown target velocity. When addressing model uncertainties and disturbances, disturbance observations were used to estimate disturbances to complete robust tracking control [32], and the NN was used to process unknown nonlinear functions, which were combined with model uncertainties and unknown external disturbances [20–23]. When the NN approximates a nonlinear function, the number of neurons has a huge impact on the error of the NN approximation function. In [33, 34], the number of neurons was very large, and the more neurons there were, the better the approximations of the nonlinear function. However, this change also led to an increase in the number of geometric series in the calculation and a drastic reduction in the calculation speed. In [35], the adaptive NN compensated for the uncertainty of the model, which used the proposed self-structure mechanism to optimize the approximation performance and reduce the computational burden. In [36], a flexible NN structure was proposed to solve the unknown nonlinear function for each neuron of multiple agents. The NN with better performance obtained by optimizing the structure was more suitable for practical application scenarios.

Inspired by the above observations and research, this paper proposes a robust target-tracking control method and a self-structuring NN strategy to solve the problems of model uncertainties and unmeasurable tracking target velocity while ensuring satisfactory USV system performance. Compared with the previous studies described in [27, 28, 37], the proposed control method is based on the fact that the speed of the tracking target cannot be obtained. In addition, for the target tracker differential explosion problem, a second-order linear differentiator is added to generate a smooth motion profile curve. In [38], the problem of input saturation is solved by introducing a Gaussian error function to avoid the output fault of the actuator. In this paper, another method is proposed to design a predefined bounded control law to guarantee that the system is ISS, to achieve input boundedness, and to guarantee that the controller is not complex. In [21, 33, 34], the use of an adaptive NN to approximate unknown model parameters required a large number of neurons to ensure the approximation effect. Then, a self-structuring neural network (SNN) optimization strategy was proposed to require fewer neurons to obtain the optimized NN structure and reduce the computational burden. In our previous work on fully actuated surface vessels [35], the SNN was first proposed to approximate the model uncertainties. However, SNNs can complete the approximation process only by adding neurons because the controller design of fully actuated surface vessels is simpler. In this paper, since the control design of underactuated surface vessels is more complex, a neural network is required to achieve higher approximation performance. Therefore, in this paper, SNNs not only can increase the number of neurons but also can delete neurons with low activation to reduce the amount of neural network training calculation on the premise of ensuring approximation performance.

The primary contributions of this paper are summarized as follows:

1. An expanded state observer is employed to estimate the nonlinear term including the target speed information so that the designed controller does not require the direct target's speed, which is very difficult to obtain in practice. In addition, the designed controller only requires the measurements of the LOS range and angle, which can receive data through some simple sensors. This ability is desirable in practice.
2. An adaptive self-structuring NN is proposed to approximate the vessel's unknown nonlinear terms, including the model uncertainties and external unknown disturbances. Compared with the RBF neural network, which has a fixed number of neurons [33, 34, 39], a self-structure strategy is developed to adjust the NN structure. This approach can optimize the NN approximation performance by adjusting the number of effective neurons, effectively reducing the computational burden.
3. Compared with other adaptive control algorithms [18], the proposed control laws are predefined as bounded and with an a priori bound, which effectively avoids input saturation of the controller.

The organizational structure of this paper is as follows.  Section 2 introduces the preparation of the USV problem formula, NN, and neuron optimization strategy.  Section 3 shows the design of the USV robust target-tracking controller and the stability analysis.  Section 4 analyses the effectiveness of the control method through simulation. Finally, Section 5 provides conclusions and future research.

## 2. Preliminaries and Problem Formulations

### 2.1. Preliminaries

Notation: *λ*_max_(·) and *λ*_min_(·) represent the largest and smallest eigenvalues of the square matrix (·), |·| denotes the absolute value of a scalar, ‖·‖ stands for the Euclidean norm, diag{·} denotes a block-diagonal matrix, and sgn(·) is a sign function.

**Assumption 1 .**

(see [40]). The matrix of the ideal NN weights is always bounded, where *W*^*∗*^ and *S*^*∗*^ are unknown positive constants that satisfy ‖*W*‖ ≤ *W*^*∗*^ and ‖*S*‖ ≤ *S*^*∗*^. *σ*_*u*_ and *σ*_*r*_ are the approximate errors, which are bounded by $\left|\sigma_{i}\right|\leq \bar{\sigma }$, *i*=*u*, *r*, and $\bar{\sigma }$ is an unknown and small positive constant.

**Assumption 2 .**

The external disturbance *d*_*w*_=[*d*_*u*_, *d*_*v*_, *d*_*r*_]^*T*^ is unmeasurable and time-varying but bounded, and its first derivative is also bounded, such that |*d*_*w*_| ≤ *d*_*w*_^*∗*^ and $\left|{\dot{d}}_{w}\right|\leq d_{wn}^{*}$, where *d*_*w*_^*∗*^ and *d*_*wn*_^*∗*^ are unknown positive constants.

### 2.2. Neural Network

Faced with the unknown dynamic model, an SNN is proposed. Suppose that *f*(*x*) : *ℝ*^*N*^⟶*ℝ* is an unknown smooth and bounded nonlinear function and that it can be approximately expressed as follows [41]:

(1) $$\begin{array}{c} f\left(x\right)=W^{T}S\left(x\right)+\sigma , \end{array}$$

where *N* is the number of neurons in the NN. *W* ∈ *ℝ*^*N*^ denotes the ideal weight vector:

(2) $$\begin{array}{c} W=\arg\min\left\{\underset{x\in \mathbb{R}}{\sup}\left|f\left(x\right)-{\hat{W}}^{T}S\left(x\right)\right|\right\}, \end{array}$$

where $\hat{W}$ is the estimation of *W*. *S*(*x*)=[*S*_1_(*x*),…,*S*_*N*_(*x*)]^*T*^ denotes the NN vector, and the activation function is a Gaussian function.

(3) $$\begin{array}{c} S_{i}\left(x\right)=\exp\left(-\frac{{\left\|x-c_{i}\right\|}^{2}}{b_{i}^{2}}\right),\;i=1,\ldots ,N, \end{array}$$

where *c*_*i*_ ∈ *ℝ*^*m*^ represents the center vector and *b*_*i*_ ∈ *ℝ* represents the width of the Gaussian function. *σ* is the bounded approximation error of the NN, namely, $\left|\sigma \right|\leq \bar{\sigma }$, and $\bar{\sigma }$ is an unknown and small constant.

In the traditional RBFNN, additional neurons in the NN result in a more accurate approximation [33, 34]. However, in actual function approximation, not all neurons are valid NN neurons. More NN neurons mean more valid as well as invalid neurons, but the former is more frequent than the latter. The SNN has the ability to increase and decrease the number of NN neurons online to achieve the best NN structure. By increasing the number of effective active neurons and deleting neurons with lower activation degrees, better function approximation performance is obtained.

The SNN neuron strategy has two principal operations: split and delete. Splitting of neurons is achieved by judging whether the neuron with the highest activation function among the existing neurons is greater than a given activation value. The maximum degree *S*_max_ among *S*_*κ*_ is defined as follows:

(4) $$\begin{array}{c} S_{\max}=\underset{1\leq \kappa \leq N}{\max}S_{\kappa }. \end{array}$$

The activation strength *S* obtained from (1) is used as the degree measure, and *S*_max_ is defined as the maximum degree among *S*_*κ*_. If *S*_*k*_ ≤ *G*_th_ where *G*_th_ ∈ (0,1) is a preset threshold, the incoming data are not ideal. In other words, the activation degree is insufficient. Therefore, a new neuron with a strong degree of activation should be split. The weight vector W and the center vector *c* corresponding to the activation function of the new neuron are the same as the parameters corresponding to the *S* neuron. This relationship ensures that the activation strength of the new split neuron is better.

The newly divided neuron is labeled as *k*^New^. The new neuron weight parameters are as follows:

(5) $$\begin{array}{c} \left\{\begin{array}{c} c_{j}^{\text{New}}=\frac{x_{j}+c_{j}}{2},\\ b_{j}^{\text{New}}=b_{j},\\ W_{j}^{\text{New}}=0,\\ I_{j}^{\text{New}}=1, \end{array}\right. \end{array}$$

where *x*_*j*_, *c*_*j*_, and *b*_*j*_ are the parameters of the largest activated neuron *S*_max_, *W*_*j*_^New^ is the initial weight value of the new neuron, and *I*_*j*_^New^ is the flag value used in (6).

If the number of neurons continues to increase, a myriad of computational pressures will be caused; therefore, the strategy of neuron deletion is proposed. When the *r* th activation strength *S*_*r*_ is smaller than a threshold *P*_th_, neuron *r* is not strongly associated with the input. Then, when *S*_*r*_ satisfies our setting strategy of continuous neuron deletion, the value of the *S*_*r*_ reference index gradually decreases. The referring index is as follows:

(6) $$\begin{array}{c} I_{r}=\left\{\begin{array}{cc} \exp\left(-\varsigma \right)I_{r}^{p} & \text{if }S_{r}\leq P_{\text{th}}\\ I_{r}^{p} & \text{if }S_{r}>P_{\text{th}} \end{array}\right.,\;r=1,2,\ldots ,N, \end{array}$$

where *I*_*r*_ is the reference index of the *r* th neuron, and its initial value is 1. *P*_th_ is the critical value for deletion, and *ς* is a positive constant. *I*_*r*_^*p*^ denotes that the final value of *I*_*r*_. *I*_th_ is a predefined value. If it satisfies *I*_*r*_ ≤ *I*_th_, the *r* th neuron is pruned. Moreover, the amount of calculation is also reduced. In summary, a neuron adjustment schematic diagram is shown in Figure 1. If *S*_*j*_ ≤ *G*_th_, a new neuron *S*_*j*_′=*S*_max_ with a strong degree of activation should be split. If inequality (6) is satisfied, the neuron is deleted. The SNN neuron algorithm strategy flowchart is shown in Figure 2.

**Remark 1 .**

The difference between RBFNN and SNN is that the former requires more neurons but introduces more low-effect neurons, which introduces a large number of invalid calculations; the latter can increase the number of effective neurons and delete inefficient neurons by judging the neurons' activation degree.

**Remark 2 .**

If the nonlinear function approximated by the SNN is more complicated, more neurons are split to obtain better approximation performance. Then, by choosing a larger *G*_th_ value, more neurons are generated, and at the same time, by slightly increasing the *P*_th_ value, activation neurons with lower degrees can be removed.

### 2.3. Problem Formulation

The kinematics and dynamics model of USVs with disturbances are expressed as follows [42]:

(7) $$\begin{array}{c} \left\{\begin{array}{c} \dot{x}=u\cos\psi -v\sin\psi ,\\ \dot{y}=u\sin\psi +v\cos\psi ,\\ \dot{\psi }=r, \end{array}\right. \end{array}$$

(8) $$\begin{array}{c} \left\{\begin{array}{c} \dot{u}=\frac{\left(F_{u}\left(u,v,r\right)+\tau_{u}+d_{u}\left(t\right)\right)}{m_{11}},\\ \dot{v}=\frac{\left(F_{v}\left(u,v,r\right)+d_{v}\left(t\right)\right)}{m_{22}},\\ \dot{r}=\frac{\left(F_{r}\left(u,v,r\right)+\tau_{r}+d_{r}\left(t\right)\right)}{m_{33}}. \end{array}\right. \end{array}$$

*η*=[*x*, *y*, *ψ*]^*T*^ represents the vessel position and orientation in the earth-fixed frame.*ν*=[*u*, *v*, *r*]^*T*^ denotes the corresponding velocities in surge, sway, and yaw. *τ*_*u*_ and *τ*_*r*_ are the control inputs. *m*_11_, *m*_22_, and *m*_33_ are the mass of the ship. *d*_*w*_=[*d*_*u*_, *d*_*v*_, *d*_*r*_]^*T*^ is an external unknown disturbance vector caused by wind, waves, and ocean currents. *F*_*j*_(*u*, *v*, *r*) (*j*=*u*, *v*, *r*) are the nonlinear function component of the ship's model, including the centripetal force and force of the Coriolis as well as the hydrodynamic damping effects and unknown dynamic model.

The target model is as follows:

(9) $$\begin{array}{c} \left\{\begin{array}{c} {\dot{x}}_{d}=u_{d}\cos\psi_{d}-v_{d}\sin\psi_{d},\\ {\dot{y}}_{d}=u_{d}\sin\psi_{d}+v_{d}\cos\psi_{d},\\ {\dot{\psi }}_{d}=\;r_{d}. \end{array}\right. \end{array}$$

A system composed of the structural relationship between the target, and the follower is shown in Figure 3.

The LOS range *z*_*e*_ and angle *ψ*_*n*_ between the target and the followers are expressed as follows:

(10) $$\begin{array}{c} \left\{\begin{array}{c} z_{e}=\sqrt{x_{e}^{2}+y_{e}^{2}},\\ \psi_{n}=a\tan2\left(y_{e},x_{e}\right), \end{array}\right. \end{array}$$

where *x*_*e*_=*x*_*d*_ − *x*, *y*_*e*_=*y*_*d*_ − *y*, and the formation tracking errors are defined by

(11) $$\begin{array}{c} \left\{\begin{array}{c} z_{d}=z_{e}-z_{n},\\ z_{\psi }=\psi_{n}-\psi -\varphi , \end{array}\right. \end{array}$$

where *z*_*n*_ is the desired LOS range and *φ*=*a*tan2(*v*, *u*) is the sideslip angle.

The control objective of this paper is to construct a robust controller for USVs (dynamics (7) and (8)) to track the desired leader trajectory so that the signals *x*_*e*_, *y*_*e*_, *z*_*d*_, and *z*_*ψ*_ are uniformly ultimately bounded (UUB).

## 3. Main Results

### 3.1. Kinematic Controller Design

The time derivatives of (11) along (9) and (7) are given by

(12) $$\begin{array}{c} \left\{\begin{array}{c} {\dot{z}}_{d}={ϒ}_{d}\left(\cdot \right)-u,\\ {\dot{z}}_{\psi }={ϒ}_{\psi }\left(\cdot \right)-r, \end{array}\right. \end{array}$$

where

(13) $$\begin{array}{c} \left\{\begin{array}{c} {ϒ}_{d}\left(\cdot \right)=u_{d}\cos\left(\psi_{n}-\psi_{d}\right)+v_{d}\sin\left(\psi_{n}-\psi_{d}\right)-v\sin\left(\psi_{n}-\psi \right)+u-u\cos\left(\psi_{n}-\psi \right)-{\dot{z}}_{n},\\ {ϒ}_{\psi }\left(\cdot \right)=\frac{\left[u_{d}\sin\left(\psi_{n}-\psi_{d}\right)+v_{d}\cos\left(\psi_{n}-\psi_{d}\right)-v\cos\left(\psi_{n}-\psi \right)+u\sin\left(\psi_{n}-\psi \right)\right]}{z_{e}}-\dot{\varphi }. \end{array}\right. \end{array}$$

**Remark 3 .**

To facilitate the derivation of the control law, coordinate transformation (11) is used, and the kinematics model of USV is rewritten as in (12). Similar error transformations are used in [42, 43].

We make the following assumptions.

**Assumption 3 .**

For the function ϒ_*d*_(*u*_*d*_, *v*_*d*_, *ψ*_*d*_, *u*, *v*, *ψ*, *ψ*_*n*_, *z*_*n*_) and ϒ_*ψ*_(*u*_*d*_, *v*_*d*_, *ψ*_*d*_, *u*, *v*, *ψ*, *ψ*_*n*_, *φ*), ϒ_*d*_^*∗*^ and ϒ_*ψ*_^*∗*^ are two positive constants, such that $\left|{\dot{ϒ}}_{d}\right|\leq {ϒ}_{d}^{*}$ and $\left|{\dot{ϒ}}_{\psi }\right|\leq {ϒ}_{\psi }^{*}$.

The kinematic controller is designed according to the error dynamics in (12). Since *u*_*d*_ and *v*_*d*_ are unknown, ϒ_*d*_ and ϒ_*ψ*_ are unavailable. Two ESOs are used to estimate ϒ_*d*_ and ϒ_*ψ*_ as follows:

(14) $$\begin{array}{c} \left\{\begin{array}{c} {\dot{\hat{z}}}_{d}=-\zeta_{1}\left({\hat{z}}_{d}-z_{d}\right)+{\hat{ϒ}}_{d}-u,\\ {\dot{\hat{ϒ}}}_{d}=-\zeta_{2}\left({\hat{z}}_{d}-z_{d}\right),\\ {\dot{\hat{z}}}_{\psi }=-\zeta_{3}\left({\hat{z}}_{\psi }-z_{\psi }\right)+{\hat{ϒ}}_{\psi }-r,\\ {\dot{\hat{ϒ}}}_{\psi }=-\zeta_{4}\left({\hat{z}}_{\psi }-z_{\psi }\right), \end{array}\right. \end{array}$$

where *ζ*_1_, *ξ*_2_, *ζ*_3_, and *ζ*_4_ are parameters that need to be designed.

The observation errors can be expressed as follows:

(15) $$\begin{array}{c} \left\{\begin{array}{c} {\dot{\tilde{z}}}_{d}=-\zeta_{1}{\tilde{z}}_{d}+{\tilde{ϒ}}_{d},\\ {\dot{\tilde{ϒ}}}_{d}=-\zeta_{2}{\tilde{z}}_{d}-{\dot{ϒ}}_{d},\\ {\dot{\tilde{z}}}_{\psi }=-\zeta_{3}{\tilde{z}}_{\psi }+{\tilde{ϒ}}_{\psi },\\ {\dot{\tilde{ϒ}}}_{\psi }=-\zeta_{4}{\tilde{z}}_{\psi }-{\dot{ϒ}}_{\psi }, \end{array}\right. \end{array}$$

where ${\tilde{z}}_{d}={\hat{z}}_{d}-z_{d}$, ${\tilde{ϒ}}_{d}={\hat{ϒ}}_{d}-{ϒ}_{d}$, ${\tilde{z}}_{\psi }={\hat{z}}_{\psi }-z_{\psi }$, and ${\tilde{ϒ}}_{\psi }={\hat{ϒ}}_{\psi }-{ϒ}_{\psi }$. Let $\tilde{H}={\left[{\tilde{z}}_{d},{\tilde{z}}_{\psi },{\tilde{ϒ}}_{d},{\tilde{ϒ}}_{\psi }\right]}^{T}$ and $\dot{ϒ}={\left[0,0,{\dot{ϒ}}_{d},{\dot{ϒ}}_{\psi }\right]}^{T}$, where $\left\|\dot{ϒ}\right\|\leq R^{*}$ and *R*^*∗*^ is a positive constant. Formula (15) is expressed as follows:

(16) $$\begin{array}{c} \dot{\tilde{H}}=\Lambda \tilde{H}-\dot{ϒ}, \end{array}$$

where Λ is a Hurwitz matrix, which is expressed as follows:

(17) $$\begin{array}{c} \Lambda =\left[\begin{array}{cccc} -\zeta_{1} & 0 & 1 & 0\\ 0 & -\zeta_{3} & 0 & 1\\ -\zeta_{2} & 0 & 0 & 0\\ 0 & -\zeta_{4} & 0 & 0 \end{array}\right]. \end{array}$$

There is a matrix P with a unique positive definite that causes the following equation to be true.

(18) $$\begin{array}{c} \Lambda^{T}P+P^{T}\Lambda =-I. \end{array}$$

Two types of virtual control laws are proposed to stabilize ${\hat{z}}_{d}$ and ${\hat{z}}_{\psi }$ as follows:

(19) $$\begin{array}{c} \left\{\begin{array}{c} \alpha_{u}=\frac{\varepsilon_{1}{\hat{z}}_{d}}{\Xi_{d}}+{\hat{ϒ}}_{d}-{\hat{e}}_{u},\\ \alpha_{r}=\frac{\varepsilon_{2}{\hat{z}}_{\psi }}{\Xi_{\psi }}+{\hat{ϒ}}_{\psi }-{\hat{e}}_{r}, \end{array}\right. \end{array}$$

where $\Xi_{d}=\sqrt{{\hat{z}}_{d}^{2}+\Omega_{d}^{2}}$ and $\Xi_{\psi }=\sqrt{{\hat{z}}_{\psi }^{2}+\Omega_{\psi }^{2}}$. Ω_*d*_ and Ω_*ψ*_ are positive parameters. *ε*_1_ and *ε*_2_ are control gain parameters. *e*_*u*_ and *e*_*r*_ are the error estimations of the tracking trajectory and angle, respectively.

Let *α*_*u*_ and *α*_*r*_ pass by the second-order linear TD to obtain *u*_*r*_ and *r*_*r*_, which are the expected values of *u* and *r*, respectively.

(20) $$\begin{array}{c} \left\{\begin{array}{c} {\dot{u}}_{r}=u_{r}^{r}m\\ {\dot{u}}_{r}^{r}=-l^{2}\left(u_{r}-\alpha_{u}\right)-2lu_{r}^{r},\\ {\dot{r}}_{r}=r_{r}^{r},\\ {\dot{r}}_{r}^{r}=-l^{2}\left(r_{r}-\alpha_{r}\right)-2lr_{r}^{r}, \end{array}\right. \end{array}$$

where *p*_*u*_=*u*_*r*_ − *α*_*u*_ and *p*_*r*_=*r*_*r*_ − *α*_*r*_. *p*_*u*_ and *p*_*r*_ are defined as estimation errors. *l* is the design parameter. The convergence of the error is analyzed in [44]; it can summarize that there exist two small positive numbers *p*_*u*_^*∗*^ and *p*_*r*_^*∗*^ that satisfy |*p*_*u*_| ≤ *p*_*u*_^*∗*^ and |*p*_*r*_| ≤ *p*_*r*_^*∗*^ for bounded virtual control signals ${\dot{\alpha }}_{u}$ and ${\dot{\alpha }}_{r}$, respectively. Then exist positive small numbers *a*_*u*_^*∗*^ and *a*_*r*_^*∗*^, such that $\left|{\dot{\alpha }}_{u}\right|\leq a_{u}^{*}$ and $\left|{\dot{\alpha }}_{r}\right|\leq a_{r}^{*}$.

Substituting (20) into (15), the target-tracking errors can be rewritten as follows:

(21) $$\begin{array}{c} \left\{\begin{array}{c} {\dot{\hat{z}}}_{d}=\frac{-\varepsilon_{1}{\hat{z}}_{d}}{\Xi_{d}}-\zeta_{1}{\tilde{z}}_{d}+{\tilde{e}}_{u}-p_{u},\\ {\dot{\hat{z}}}_{\psi }=\frac{-\varepsilon_{2}{\hat{z}}_{\psi }}{\Xi_{\psi }}-\zeta_{3}{\tilde{z}}_{\psi }+{\tilde{e}}_{r}-p_{r}, \end{array}\right. \end{array}$$

where *e*_*u*_=*u* − *u*_*r*_, *e*_*r*_=*r* − *r*_*r*_, ${\tilde{e}}_{u}={\hat{e}}_{u}-e_{u}$, and ${\tilde{e}}_{r}={\hat{e}}_{r}-e_{r}$.

### 3.2. Dynamic Controller Design

From equation (8), the derivatives of *e*_*u*_ and *e*_*r*_ are expressed as follows:

(22) $$\begin{array}{c} \left\{\begin{array}{c} m_{11}{\dot{e}}_{u}={\bar{F}}_{u}\left(\cdot \right)+\tau_{u},\\ m_{33}{\dot{e}}_{r}={\bar{F}}_{r}\left(\cdot \right)+\tau_{r}, \end{array}\right. \end{array}$$

where ${\bar{F}}_{u}\left(\cdot \right)=F_{u}\left(u,v,r\right)+d_{u}-m_{11}{\dot{u}}_{r}$ and ${\bar{F}}_{r}\left(\cdot \right)=F_{r}\left(u,v,r\right)+d_{r}-m_{33}{\dot{r}}_{r}$. ${\bar{F}}_{u}\left(\cdot \right)$ and ${\bar{F}}_{r}\left(\cdot \right)$ are the unknown nonlinear function components of the ship's model and the unknown external disturbances. In the process of deriving the control law, it is necessary to solve the nonlinear function, which is composed of unknown disturbances and uncertainties from the model. Inspired by the SNN, a parameter adaptive method is proposed to approximate nonlinear functions ${\bar{F}}_{u}\left(\cdot \right)$ and ${\bar{F}}_{r}\left(\cdot \right)$.

(23) $$\begin{array}{c} \left\{\begin{array}{c} {\bar{F}}_{u}=W_{u}^{T}S_{u}\left(Z\right)+\sigma_{u},\\ {\bar{F}}_{r}=W_{r}^{T}S_{r}\left(Z\right)+\sigma_{r}, \end{array}\right. \end{array}$$

where $Z={\left[{\dot{u}}_{r},{\dot{r}}_{r},e_{u},e_{r}\right]}^{T}\in {\mathbb{R}}^{4}$ is the input vector and *S*_*u*_(*Z*) and *S*_*r*_(*Z*) are the RBF vectors. *σ*_*u*_ and *σ*_*r*_ are the approximate errors, which are bounded. *W*_*u*_ and *W*_*r*_ denote the ideal weights. ${\hat{W}}_{u}$ and ${\hat{W}}_{r}$ are the estimation values of *W*_*u*_ and *W*_*r*_, respectively. *W*_*u*_^*∗*^, *W*_*r*_^*∗*^, *S*_*u*_^*∗*^, and *S*_*r*_^*∗*^ are unknown positive constants that satisfy ‖*W*_*u*_‖ ≤ *W*_*u*_^*∗*^, ‖*W*_*r*_‖ ≤ *W*_*r*_^*∗*^, ‖*S*_*u*_‖ ≤ *S*_*u*_^*∗*^, and ‖*S*_*u*_‖ ≤ *S*_*u*_^*∗*^, respectively.

Error estimation models are designed based on the SNN as follows:

(24) $$\begin{array}{c} \left\{\begin{array}{c} m_{11}{\dot{\hat{e}}}_{u}={\hat{W}}_{u}^{T}S_{u}\left(Z\right)+\tau_{u}-\left(\varepsilon_{3}+\delta_{u}\right){\tilde{e}}_{u},\\ m_{33}{\dot{\hat{e}}}_{r}={\hat{W}}_{r}^{T}S_{r}\left(Z\right)+\tau_{r}-\left(\varepsilon_{4}+\delta_{r}\right){\tilde{e}}_{r}, \end{array}\right. \end{array}$$

where *ε*_3_, *ε*_4_, *δ*_*u*_, and *δ*_*r*_ are the positive constant parameters.

Then, the control laws based on the SNN models (24) are designed as follows:

(25) $$\begin{array}{c} \left\{\begin{array}{c} \tau_{u}=\frac{-\varepsilon_{3}{\hat{e}}_{u}}{\Xi_{u}}-{\hat{W}}_{u}^{T}S_{u}\left(Z\right),\\ \tau_{r}=\frac{-\varepsilon_{4}{\hat{e}}_{r}}{\Xi_{r}}-{\hat{W}}_{r}^{T}S_{r}\left(Z\right), \end{array}\right. \end{array}$$

where $\Xi_{u}=\sqrt{{\hat{e}}_{u}^{2}+\Omega_{u}^{2}}$, $\Xi_{r}=\sqrt{{\hat{e}}_{r}^{2}+\Omega_{r}^{2}}$, and Ω_*u*_ and Ω_*r*_ are two positive constants. Design the following adaptive update laws for ${\hat{W}}_{u}$ and ${\hat{W}}_{r}$ as follows:

(26) $$\begin{array}{c} \left\{\begin{array}{c} {\dot{\hat{W}}}_{u}=-\Gamma_{u}\left(S_{u}\left(Z\right){\hat{e}}_{u}+\rho_{1}{\hat{W}}_{u}\right),\\ {\dot{\hat{W}}}_{r}=-\Gamma_{r}\left(S_{r}\left(Z\right){\hat{e}}_{r}+\rho_{2}{\hat{W}}_{r}\right), \end{array}\right. \end{array}$$

where Γ_*u*_, Γ_*r*_, *ρ*_1_, and *ρ*_2_ are the design parameters.

**Remark 4 .**

The estimation errors ${\hat{e}}_{u}$ are used to replace the errors *e*_*u*_, which effectively improves the transient performance of the control system [45].

The designed control laws (25) are bounded, and the bound are a priori, which effectively avoids saturation of the controller. The upper bound of the control laws can be expressed as follows:

(27) $$\begin{array}{c} \left\{\begin{array}{c} \left|\tau_{u}\right|\leq \varepsilon_{3}+W_{u}^{*}S_{u}^{*},\\ \left|\tau_{r}\right|\leq \varepsilon_{4}+W_{r}^{*}S_{r}^{*}. \end{array}\right. \end{array}$$

**Remark 5 .**

The SNN weights *W*_*u*_ ∈ *ℝ*^*L*^ and *W*_*r*_ ∈ *ℝ*^*L*^ are trained and self-learned online according to (26). *L* is the number of neurons in the SNN, which can be updated according to the self-structuring strategy.

Substituting (25) into (24) yields

(28) $$\begin{array}{c} \left\{\begin{array}{c} m_{11}{\dot{\hat{e}}}_{u}=\frac{-\varepsilon_{3}{\hat{e}}_{u}}{\Xi_{u}}-\left(\varepsilon_{3}+\delta_{u}\right){\tilde{e}}_{u},\\ m_{33}{\dot{\hat{e}}}_{r}=\frac{-\varepsilon_{4}{\hat{e}}_{r}}{\Xi_{r}}-\left(\varepsilon_{4}+\delta_{r}\right){\tilde{e}}_{r}. \end{array}\right. \end{array}$$

The derivatives of ${\tilde{W}}_{u}$, ${\tilde{W}}_{r}$, ${\tilde{e}}_{u}$, and ${\tilde{e}}_{r}$ along (26) and (24) are as follows:

(29) $$\begin{array}{c} \left\{\begin{array}{c} {\dot{\tilde{W}}}_{u}=-\Gamma_{u}\left(S_{u}\left(Z\right){\hat{e}}_{u}+\rho_{1}{\hat{W}}_{u}\right),\\ {\dot{\tilde{W}}}_{r}=-\Gamma_{r}\left(S_{r}\left(Z\right){\hat{e}}_{r}+\rho_{2}{\hat{W}}_{r}\right),\\ m_{11}{\dot{\tilde{e}}}_{u}=-\left(\varepsilon_{3}+\delta_{u}\right){\tilde{e}}_{u}+{\tilde{W}}_{u}^{T}S_{u}\left(Z\right)-\sigma_{u},\\ m_{33}{\dot{\tilde{e}}}_{r}=-\left(\varepsilon_{4}+\delta_{r}\right){\tilde{e}}_{r}+{\tilde{W}}_{r}^{T}S_{r}\left(Z\right)-\sigma_{r}, \end{array}\right. \end{array}$$

where ${\tilde{W}}_{u}={\hat{W}}_{u}-W_{u}$ and ${\tilde{W}}_{r}={\hat{W}}_{r}-W_{r}$ are the estimation errors. The control scheme flow is shown in Figure 4.

### 3.3. Stability Analysis

The closed-loop error system is a cascade system composed of two estimation error subsystems ((16) and (29)) and a target-tracking error subsystem ((21) and (28)). Three lemmas are used to prove its stability. The first is the stability of the ESOs observation error system.

**Lemma 1 .**

There is a matrix *P* with a positive definite that satisfies (18), and the error system in (16) is a system for which the state is $\tilde{H}$ and the input is $\dot{ϒ}$. Then, the error system (16) is input-to-state stable (ISS) under Assumption 3.

**Proof**

Define the Lyapunov function concerned with ESOs error as follows:

(30) $$\begin{array}{c} V_{1}=\frac{1}{2}{\tilde{H}}^{T}P\tilde{H}. \end{array}$$

The time derivative of *V*_1_ along (18) becomes

(31) $$\begin{array}{c} {\dot{V}}_{1}={\tilde{H}}^{T}\left(\Lambda^{T}P+P^{T}\Lambda \right)\tilde{H}+{\tilde{H}}^{T}P\left(-\dot{ϒ}\right)\leq -{\left\|\tilde{H}\right\|}^{2}+\left\|\tilde{H}\right\|\left\|P\right\|\left\|\dot{ϒ}\right\|. \end{array}$$

Since

(32) $$\begin{array}{c} \left\|\tilde{H}\right\|\geq \frac{\left\|P\right\|\left\|\dot{ϒ}\right\|}{\mu_{1}} \end{array}$$

renders

(33) $$\begin{array}{c} {\dot{V}}_{1}\leq -\left(1-\mu_{1}\right){\left\|\tilde{H}\right\|}^{2}, \end{array}$$

where 0 < *μ*_1_ < 1, it follows that the observer error system is ISS, and

(34) $$\begin{array}{c} \left\|\tilde{H}\left(t\right)\right\|\leq \max\left\{\beta_{1}\left(\left\|\tilde{H}\left(0\right)\right\|,t\right),\gamma^{\dot{ϒ}}\left(\left\|\dot{ϒ}\right\|\right)\right\}, \end{array}$$

where *β*_1_ is a *𝒦*ℒ function and

(35) $$\begin{array}{c} \gamma^{\dot{ϒ}}\left(r\right)=\sqrt{\frac{\lambda_{\max}\left(P\right)}{\lambda_{\min}\left(P\right)}}\frac{\left\|P\right\|r}{\mu_{1}}. \end{array}$$

Then, the stability of the error subsystem (24) is given by Lemma 2.

**Lemma 2 .**

The error subsystem (24), considered as a system with the inputs being *σ*_*u*_, *σ*_*r*_, ${\tilde{W}}_{u}$, and ${\tilde{W}}_{r}$ and the states being ${\tilde{e}}_{u}$, ${\tilde{e}}_{r}$, ${\tilde{W}}_{u}$, and ${\tilde{W}}_{r}$, is ISS under Assumption 1.

**Proof**

Assign the Lyapunov function as follows:

(36) $$\begin{array}{c} V_{2}=\frac{1}{2}m_{11}{\tilde{e}}_{u}^{2}+\frac{1}{2}m_{33}{\tilde{e}}_{r}^{2}+\frac{1}{2}{\tilde{W}}_{u}^{T}\Gamma_{u}^{-1}{\tilde{W}}_{u}+\frac{1}{2}{\tilde{W}}_{r}^{T}\Gamma_{r}^{-1}{\tilde{W}}_{r}. \end{array}$$

With (29), the derivative of (36) is as follows:

(37) $$\begin{array}{c} {\dot{V}}_{2}={\tilde{e}}_{u}m_{11}{\dot{\tilde{e}}}_{u}+{\tilde{e}}_{r}m_{11}{\dot{\tilde{e}}}_{r}+{\tilde{W}}_{u}^{T}\Gamma_{u}^{-1}{\dot{\hat{W}}}_{u}+{\tilde{W}}_{r}^{T}\Gamma_{r}^{-1}{\dot{\hat{W}}}_{r}\\ =-\left(\varepsilon_{3}+\delta_{u}\right){\tilde{e}}_{u}^{2}-\sigma_{u}{\tilde{e}}_{u}-\left(\varepsilon_{4}+\delta_{r}\right){\tilde{e}}_{r}^{2}-\sigma_{r}{\tilde{e}}_{r}-\rho_{1}{\left\|{\tilde{W}}_{u}\right\|}^{2}-\rho_{1}\left\|{\tilde{W}}_{u}\right\|\left\|W_{u}\right\|-\rho_{2}{\left\|{\tilde{W}}_{r}\right\|}^{2}-\rho_{2}\left\|{\tilde{W}}_{r}\right\|\left\|W_{u}\right\|\\ =-X_{1}^{T}E_{1}X_{1}+l_{1}^{T}X_{1}, \end{array}$$

where ${Χ}_{1}={\left[{\tilde{e}}_{u},{\tilde{e}}_{r},\left\|{\tilde{W}}_{u}\right\|,\left\|{\tilde{W}}_{r}\right\|\right]}^{T}$, *E*_1_=diag{*ε*_3_+*δ*_*u*_, *ε*_4_+*δ*_*r*_, *ρ*_1_, *ρ*_2_}, and *l*_1_=[−*σ*_*u*_, −*σ*_*r*_, *ρ*_1_‖*W*_*u*_‖, *ρ*_2_‖*W*_*r*_‖]^*T*^.

Since

(38) $$\begin{array}{c} \left\|{Χ}_{1}\right\|\geq \frac{\left\|l_{1}\right\|}{\mu_{2}\lambda_{\min}\left(E_{1}\right)}\\ \geq \frac{\left|\sigma_{u}\right|}{\mu_{2}\lambda_{\min}\left(E_{1}\right)}+\frac{\left|\sigma_{r}\right|}{\mu_{2}\lambda_{\min}\left(E_{1}\right)}+\frac{\left|\rho_{1}\right|\left\|W_{u}\right\|}{\mu_{2}\lambda_{\min}\left(E_{1}\right)}+\frac{\left|\rho_{2}\right|\left\|W_{r}\right\|}{\mu_{2}\lambda_{\min}\left(E_{1}\right)} \end{array}$$

renders

(39) $$\begin{array}{c} {\dot{V}}_{2}\leq -\left(1-\mu_{2}\right)\lambda_{\min}\left(E_{1}\right){\left\|X_{1}\right\|}^{2}, \end{array}$$

where 0 < *μ*_2_ < 1. Consequently, the error subsystem (24) is ISS, and

(40) $$\begin{array}{c} \left\|X_{1}\left(t\right)\right\|\leq \max\left\{\beta_{2}\left(\left\|X_{1}\left(0\right)\right\|,t\right),\gamma^{\sigma_{u}}\left(\left|\sigma_{u}\right|\right)+\gamma^{\sigma_{u}}\left(\left|\sigma_{r}\right|\right)+\gamma^{W_{u}}\left(\left\|W_{u}\right\|\right)+\gamma^{W_{r}}\left(\left\|W_{r}\right\|\right)\right\}, \end{array}$$

where *β*_2_ is a *𝒦*ℒ function and

(41) $$\begin{array}{c} \left\{\begin{array}{c} \gamma^{\sigma_{u}}\left(r\right)=\sqrt{\frac{\lambda_{\max}\left(N_{1}\right)}{\lambda_{\min}\left(N_{1}\right)}}\frac{r}{\mu_{2}\lambda_{\min}\left(E_{1}\right)},\\ \gamma^{\sigma_{r}}\left(r\right)=\sqrt{\frac{\lambda_{\max}\left(N_{1}\right)}{\lambda_{\min}\left(N_{1}\right)}}\frac{r}{\mu_{2}\lambda_{\min}\left(E_{1}\right)},\\ \gamma^{W_{u}}\left(r\right)=\sqrt{\frac{\lambda_{\max}\left(N_{1}\right)}{\lambda_{\min}\left(N_{1}\right)}}\frac{\rho_{1}r}{\mu_{2}\lambda_{\min}\left(E_{1}\right)},\\ \gamma^{W_{r}}\left(r\right)=\sqrt{\frac{\lambda_{\max}\left(N_{1}\right)}{\lambda_{\min}\left(N_{1}\right)}}\frac{\rho_{2}r}{\mu_{2}\lambda_{\min}\left(E_{1}\right)}, \end{array}\right. \end{array}$$

where *N*_1_=diag{*m*_11_, *m*_33_, Γ_*u*_^−1^, Γ_*r*_^−1^}.

The last is the stability of the target-tracking error subsystems (21) and (28).

**Lemma 3 .**

Subsystems (21) and (28), considered as a system with the inputs being $\tilde{H}$, ${\tilde{e}}_{u}$, ${\tilde{e}}_{r}$, ${\tilde{p}}_{u}$, and ${\tilde{p}}_{r}$ and the states being ${\hat{e}}_{u}$, ${\hat{e}}_{r}$, ${\hat{z}}_{d}$, and ${\hat{z}}_{\psi }$, are ISS.

**Proof**

Define the Lyapunov function as follows:

(42) $$\begin{array}{c} V_{3}=\frac{1}{2}{\hat{z}}_{d}^{2}+\frac{1}{2}{\hat{z}}_{\psi }^{2}+\frac{1}{2}m_{11}{\hat{e}}_{u}^{2}+\frac{1}{2}m_{33}{\hat{e}}_{r}^{2}. \end{array}$$

Substituting (21) and (28) into the derivative of (42), the following is obtained:

(43) $$\begin{array}{c} {\dot{V}}_{3}=-\frac{\varepsilon_{1}{\hat{z}}_{d}^{2}}{\Xi_{d}}-{\hat{z}}_{d}\left(\zeta_{1}{\tilde{z}}_{d}-{\tilde{e}}_{u}+p_{u}\right)-\frac{\varepsilon_{2}{\hat{z}}_{\psi }^{2}}{\Xi_{\psi }}-{\hat{z}}_{\psi }\left(\zeta_{3}{\tilde{z}}_{\psi }-{\tilde{e}}_{r}+p_{r}\right)-\frac{\varepsilon_{3}{\hat{e}}_{u}^{2}}{\Xi_{u}}-{\hat{e}}_{u}\left(\varepsilon_{3}+\delta_{u}\right){\tilde{e}}_{u}-\frac{\varepsilon_{4}{\hat{e}}_{r}^{2}}{\Xi_{r}}-{\hat{e}}_{r}\left(\varepsilon_{4}+\delta_{r}\right){\tilde{e}}_{r}\\ \leq -\frac{\lambda_{\min}\left(E_{2}\right){\left\|X_{2}\right\|}^{2}}{\sqrt{{\left\|X_{2}\right\|}^{2}+\Omega_{\max}^{2}}}+\left\|l_{2}\right\|\left\|X_{2}\right\|, \end{array}$$

where $l_{2}={\left[\zeta_{1}\left|{\tilde{z}}_{d}\right|+\left|{\tilde{e}}_{u}\right|+\left|p_{u}\right|,\zeta_{3}\left|{\tilde{z}}_{\psi }\right|+\left|{\tilde{e}}_{r}\right|+\left|p_{r}\right|,\left(\varepsilon_{3}+\delta_{u}\right)\left|{\tilde{e}}_{u}\right|,\left(\varepsilon_{4}+\delta_{r}\right)\left|{\tilde{e}}_{r}\right|\right]}^{T}$, *E*_2_=diag{*ε*_1_, *ε*_2_, *ε*_3_, *ε*_4_}, $X_{2}={\left[{\hat{z}}_{d},{\hat{z}}_{\psi },{\hat{e}}_{u},{\hat{e}}_{r}\right]}^{T}$, and Ω_max_=max{Ω_*d*_, Ω_*ψ*_, Ω_*u*_, Ω_*r*_}.

Since

(44) $$\begin{array}{c} \frac{\left\|X_{2}\right\|}{\sqrt{{\left\|X_{2}\right\|}^{2}+\Omega_{\max}^{2}}}\geq \frac{\left\|l_{2}\right\|}{\mu_{3}\lambda_{\min}\left(E_{2}\right)}\\ \geq \frac{\zeta_{1}\left|{\tilde{z}}_{d}\right|}{\mu_{3}\lambda_{\min}\left(E_{2}\right)}+\frac{\left|p_{u}\right|}{\mu_{3}\lambda_{\min}\left(E_{2}\right)}+\frac{\zeta_{3}\left|{\tilde{z}}_{\psi }\right|}{\mu_{3}\lambda_{\min}\left(E_{2}\right)}+\frac{\left|p_{r}\right|}{\mu_{3}\lambda_{\min}\left(E_{2}\right)}+\frac{\left(1+\varepsilon_{3}+\delta_{u}\right)\left|{\tilde{e}}_{u}\right|}{\mu_{3}\lambda_{\min}\left(E_{2}\right)}+\frac{\left(1+\varepsilon_{4}+\delta_{r}\right)\left|{\tilde{e}}_{r}\right|}{\mu_{3}\lambda_{\min}\left(E_{2}\right)}, \end{array}$$

renders

(45) $$\begin{array}{c} {\dot{V}}_{3}\leq -\frac{\left(1-\mu_{3}\right)\lambda_{\min}\left(E_{2}\right){\left\|X_{2}\right\|}^{2}}{\sqrt{{\left\|X_{2}\right\|}^{2}+\Omega_{\max}^{2}}}, \end{array}$$

where 0 < *μ*_3_ < 1, it shows that subsystems (21) and (28) are ISS, and

(46) $$\begin{array}{c} \left\|X_{2}\left(t\right)\right\|\leq \max\left\{\beta_{3}\left(\left\|X_{2}\left(0\right)\right\|,t\right),\gamma^{{\tilde{z}}_{d}}\left(\left|{\tilde{z}}_{d}\right|\right)+\gamma^{p_{u}}\left(\left|p_{u}\right|\right)+\gamma^{{\tilde{z}}_{\psi }}\left(\left|{\tilde{z}}_{\psi }\right|\right)+\gamma^{p_{r}}\left(\left|p_{r}\right|\right)+\gamma^{{\tilde{e}}_{u}}\left(\left|{\tilde{e}}_{u}\right|\right)+\gamma^{{\tilde{e}}_{r}}\left(\left|{\tilde{e}}_{r}\right|\right)\right\}, \end{array}$$

where *β*_3_ is a *𝒦*ℒ function and

(47) $$\begin{array}{c} \left\{\begin{array}{c} \gamma^{{\tilde{z}}_{d}}\left(r\right)=\varpi^{-1}\sqrt{\frac{\lambda_{\max}\left(N_{2}\right)}{\lambda_{\min}\left(N_{2}\right)}}\frac{\zeta_{1}r}{\mu_{3}\lambda_{\min}\left(E_{2}\right)},\\ \gamma^{p_{u}}\left(r\right)=\varpi^{-1}\sqrt{\frac{\lambda_{\max}\left(N_{2}\right)}{\lambda_{\min}\left(N_{2}\right)}}\frac{r}{\mu_{3}\lambda_{\min}\left(E_{2}\right)},\\ \gamma^{{\tilde{z}}_{\psi }}\left(r\right)=\varpi^{-1}\sqrt{\frac{\lambda_{\max}\left(N_{2}\right)}{\lambda_{\min}\left(N_{2}\right)}}\frac{\zeta_{3}r}{\mu_{3}\lambda_{\min}\left(E_{2}\right)},\\ \gamma^{p_{r}}\left(r\right)=\varpi^{-1}\sqrt{\frac{\lambda_{\max}\left(N_{2}\right)}{\lambda_{\min}\left(N_{2}\right)}}\frac{r}{\mu_{3}\lambda_{\min}\left(E_{2}\right)},\\ \gamma^{{\tilde{e}}_{u}}\left(r\right)=\varpi^{-1}\sqrt{\frac{\lambda_{\max}\left(N_{2}\right)}{\lambda_{\min}\left(N_{2}\right)}}\frac{\left(1+\varepsilon_{3}+\delta_{u}\right)r}{\mu_{3}\lambda_{\min}\left(E_{2}\right)},\\ \gamma^{{\tilde{e}}_{r}}\left(r\right)=\varpi^{-1}\sqrt{\frac{\lambda_{\max}\left(N_{2}\right)}{\lambda_{\min}\left(N_{2}\right)}}\frac{\left(1+\varepsilon_{4}+\delta_{r}\right)r}{\mu_{3}\lambda_{\min}\left(E_{2}\right)}, \end{array}\right. \end{array}$$

with $\varpi \left(r\right)=r^{2}/\sqrt{r^{2}+\Omega_{\max}^{2}}$ and *N*_2_=diag{1, *m*_11_, *m*_33_}.

Therefore, the stability of the cascade of ESO error subsystem (16), subsystem (29), and target-tracking error subsystems (21) and (28) is given by the following theorem.

**Theorem 1 .**

The cascade system composed of ESO error subsystem (16), subsystem (29), and target-tracking error subsystems (21) and (28) is ISS under Assumptions 1, 2, and 3. And all errors of the closed-loop system are uniformly ultimately bounded.

**Proof**

Lemmas 1–3 prove that observer error subsystems (16) with input $\dot{ϒ}$ and state $\tilde{H}$; subsystems (29) with inputs *σ*_*u*_, *σ*_*r*_, ${\tilde{W}}_{u}$, and ${\tilde{W}}_{r}$ and states ${\tilde{e}}_{u}$, ${\tilde{e}}_{r}$, ${\tilde{W}}_{u}$, and ${\tilde{W}}_{r}$; and target-tracking error subsystems (21) and (28) with inputs $\tilde{H}$, ${\tilde{e}}_{u}$, ${\tilde{e}}_{r}$, ${\tilde{p}}_{u}$, and ${\tilde{p}}_{r}$ and states ${\hat{e}}_{u}$, ${\hat{e}}_{r}$, ${\hat{z}}_{d}$, and ${\hat{z}}_{\psi }$ are ISS, respectively. According to cascade stability theory (Lemma 4.6 in [46]), the closed-loop error system composed of (16), (29), and (21) and (28) is ISS with states $\tilde{H}$, ${\tilde{e}}_{u}$, ${\tilde{e}}_{r}$, ${\tilde{W}}_{u}$, and ${\tilde{W}}_{r}$; ${\hat{e}}_{u}$, ${\hat{e}}_{r}$, ${\hat{z}}_{d}$, and ${\hat{z}}_{\psi }$; and inputs $\dot{ϒ}$, *σ*_*u*_, *σ*_*r*_, ${\tilde{W}}_{u}$, ${\tilde{W}}_{r}$, ${\tilde{e}}_{u}$, ${\tilde{e}}_{r}$, ${\tilde{p}}_{u}$, and ${\tilde{p}}_{r}$. In conclusion, when *t* > 0 is satisfied, ‖*E*(*t*)‖ satisfies the inequality as follows:

(48) $$\begin{array}{c} \left\|E\left(t\right)\right\|\leq \beta \left(\left\|E\left(0\right)\right\|,t\right)+\gamma \left(\left\|\dot{ϒ},\sigma_{u},\sigma_{r},W_{u},W_{r},{\tilde{e}}_{u},{\tilde{e}}_{r},{\tilde{p}}_{u},{\tilde{p}}_{r}\right\|\right), \end{array}$$

where $E=\left[\tilde{H},{\tilde{e}}_{u},{\tilde{e}}_{r},{\tilde{W}}_{u},{\tilde{W}}_{r},{\tilde{e}}_{u},{\tilde{e}}_{r},{\hat{z}}_{d},{\hat{z}}_{\psi }\right]$. $\dot{ϒ},\sigma_{u},\sigma_{r},W_{u},W_{r},{\tilde{e}}_{u},{\tilde{e}}_{r},{\tilde{p}}_{u}$, and ${\tilde{p}}_{r}$ are bounded by *p*_*u*_^*∗*^, *p*_*r*_^*∗*^, and Assumptions 1 and 2.

As a consequence, the errors $\tilde{H}$, ${\tilde{e}}_{u}$, ${\tilde{e}}_{r}$, ${\tilde{W}}_{u}$, ${\tilde{W}}_{r}$, ${\hat{e}}_{u}$, ${\hat{e}}_{r}$, ${\hat{z}}_{d}$, and ${\hat{z}}_{\psi }$ are all bounded.

(49) $$\begin{array}{c} \left\{\begin{array}{c} \left|z_{d}\right|=\left|{\hat{z}}_{d}-{\tilde{z}}_{d}\right|\leq \left|{\hat{z}}_{d}\right|+\left|{\tilde{z}}_{d}\right|,\\ \left|z_{\psi }\right|=\left|{\hat{z}}_{\psi }-{\tilde{z}}_{\psi }\right|\leq \left|{\hat{z}}_{\psi }\right|+\left|{\tilde{z}}_{\psi }\right|,\\ \left|e_{u}\right|=\left|{\hat{e}}_{u}-{\tilde{e}}_{u}\right|\leq \left|{\hat{e}}_{u}\right|+\left|{\tilde{e}}_{u}\right|,\\ \left|e_{r}\right|=\left|{\hat{e}}_{r}-{\tilde{e}}_{r}\right|\leq \left|{\hat{e}}_{r}\right|+\left|{\tilde{e}}_{r}\right|. \end{array}\right. \end{array}$$

**Theorem 2 .**

Since ${\hat{z}}_{d}$, ${\tilde{z}}_{d}$${\hat{z}}_{\psi }$, ${\tilde{z}}_{\psi }$${\hat{e}}_{u}$, ${\tilde{e}}_{u}$, ${\hat{e}}_{r}$, and ${\tilde{e}}_{r}$ are both bounded, it means that the tracking errors *z*_*d*_, *z*_*ψ*_, *e*_*u*_, and *e*_*r*_ are all bounded.

**Remark 6 .**

Figure 5 represents the tracking relationship between leader and follower in target tracking. A formation has multiple leaders and followers, and a formation can be decomposed into many subsystems of one leader and one follower. A similar formation control structure is also available in [43]. Followers in each subsystem maintain the desired location of the target, then the desired formation is established.

## 4. Simulation Results

In this section, to verify the effectiveness of the control method, a simulation model is established. Consider a USV team with two levels of control, which consists of a tracking target and two followers. USV1 follows the target vessel, and USV2 follows USV1. The USV model parameters are shown in [10].

The unknown nonlinear function in the USV model is expressed as follows:

(50) $$\begin{array}{c} \left\{\begin{array}{c} F_{u}\left(u,v,r\right)=33.8vr-12u-2.5\left|u\right|u+g_{u},\\ F_{v}\left(u,v,r\right)=-25.8ur-0.2r-17v-4.5\left|v\right|v+g_{v},\\ F_{r}\left(u,v,r\right)=-33.8vr+25.8uv-0.5v-0.5r-0.1\left|r\right|r+g_{r}, \end{array}\right. \end{array}$$

where the unknown model uncertainties are assumed to be

(51) $$\begin{array}{c} \left\{\begin{array}{c} g_{u}=0.05v^{2}r+0.035uv^{2},\\ g_{v}=0.1u^{2}v,\\ g_{r}=0.035urv^{3}+0.032ur^{2}. \end{array}\right. \end{array}$$

The external disturbances are simulated as follows:

(52) $$\begin{array}{c} \left\{\begin{array}{c} d_{u}\left(t\right)=0.9\sin\left(0.3t\right)\cos\left(0.1t\right)+0.8\sin\left(0.2t\right)\sin\left(0.1t\right),\\ d_{v}\left(t\right)=0.1\sin\left(0.1t\right),\\ d_{r}\left(t\right)=1.1\cos\left(0.3t\right)\sin\left(0.2t\right). \end{array}\right. \end{array}$$

The position velocities of the tracking target are considered to be *u*_*d*_=0.25 and *v*_*d*_=0, and the yaw angle velocity is designed as follows:

(53) $$\begin{array}{c} \left\{\begin{array}{cc} r_{d}=-0.015, & \text{if }t\leq 210,\\ r_{d}=0.015, & \text{if }210<t\leq 630,\\ r_{d}=-0.015, & \text{if }630<t. \end{array}\right. \end{array}$$

The initial positions of the USVs and target are [−25,10,0]^*T*^ and [−30, −10,0]^*T*^. The desired LOS tracking position range is expressed as *z*_*n*1_=*z*_*n*2_=5. The control parameters of the SNN are selected as *ζ*_1_=20, *ζ*_2_=100, *ζ*_3_=20, *ζ*_4_=100, *ε*_1_=0.5, *ε*_2_=0.1, *ε*_3_=0.5, *ε*_4_=0.1, Ω_*d*_=2, Ω_*ψ*_=2, Ω_*u*_=2, Ω_*r*_=1, *l*=1.4, Γ_*u*_=40, Γ_*r*_=40, *δ*_*u*_=120, *δ*_*r*_=40, *ρ*_1_=*ρ*_2_=0.1, *G*_th_=0.9, *P*_th_=0.1, and *ς*=0.7.

The simulation results are shown in Figures 6–11.  Figure 6 shows the trajectory of the tracking target and the followers. The two ships move from different initial positions to the desired position. This result shows that the controller designed in this paper completes target-tracking control under uncertain nonlinear terms and unknown external disturbances. When both followers complete target tracking, a specific formation is achieved. The performance of the ESO is shown in Figure 7.  Figure 8 shows that the neural network fits nonlinear functions composed of unknown dynamic models and external disturbances.  Figure 9 shows the control input and its bounds.  Figure 10 shows the trend in the number of neurons in the SNN as well as the number after stabilization. In the beginning, the nonlinear function changes considerably, so the SNN must continuously split neurons and delete invalid neural neurons when approaching it. This leads to greater changes in neurons. When the SNN output approximates the nonlinear function, the number of neurons gradually stabilizes, and when the approximation performance reaches the best, the number of neurons stabilizes. The target-tracking error is shown in Figure 11, and it represents a small neighborhood where the tracking error will converge to zero.

In addition, to verify the performance of the SNN, the performances of the RBFNN and SNN using the same parameters except for the number of neurons are compared. The number of neurons in the RBFNN is *N*_1_=48 The RBFNN control parameters are selected as Γ_1*u*_=40, Γ_1*r*_=40, and *ρ*_11_=*ρ*_12_=0.1.

(54) $$\begin{array}{c} \left\{\begin{array}{c} {\dot{\hat{W}}}_{1u}=-\Gamma_{1u}\left(S_{u}\left(Z\right){\tilde{e}}_{u}+\rho_{11}{\hat{W}}_{1u}\right),\\ {\dot{\hat{W}}}_{1r}=-\Gamma_{1r}\left(S_{r}\left(Z\right){\tilde{e}}_{r}+\rho_{21}{\hat{W}}_{1r}\right). \end{array}\right. \end{array}$$

The approximation performance of the RBFNN is shown in Figure 12. The SNN and RBFNN approximation errors are shown in Figure 13. Figures 12 and 13 show that the approximate performance of the RBFNN with 48 neurons is excellent and that the approximation errors are small. In Figure 13, the approximation errors of the SNN are smaller than those of the RBFNN, demonstrating that the approximation performance of the SNN is better.  Figure 9 shows that the maximum number of SNN neurons in USV1 exceeds 28 and remains at 24. Consequently, when guaranteeing approximation performance and when the unknown nonlinear component is complicated, more neurons are needed, and when the unknown nonlinear component is simple, only a small number of neurons is needed. By optimizing the number of neurons, the approximation performance of the NN is guaranteed, and the amount of calculation is reduced.

To verify the performance of the proposed controller, a comparison with adaptive output-feedback control [18] is provided. The LOS range error, angle tracking error, and control inputs are shown in Figures 14–17. As seen in Figure 14, the proposed method's LOS range tracking error is smaller than that in [18]. In Figure 15, the angle tracking errors of the two methods are similar. As seen in Figures 16 and 17, the initial values of the control inputs *τ*_*u*_ and *τ*_*r*_ in method [18] are much larger than those of the proposed method, exceeding 600 N and 40 N•m, respectively. The control inputs are physically limited by the actuator, and exceeding the limits can cause actuator saturation, which may lead to degraded performance, hysteresis, and instability. In Figure 8, the proposed method's control inputs *τ*_*u*_ and *τ*_*r*_ are less than 15 N and 5 N•m, respectively. In conclusion, compared with the method in [18], the proposed method has smaller tracking errors and no input saturation problem.

## 5. Conclusions

In this paper, a target-tracking controller for USVs with model uncertainties and external low-frequency disturbances is proposed. The speed of the target is unknown, and only the position and angle are measured. An ESO-based motion controller is proposed, and it can estimate the unknown nonlinear function of the target caused by the unavailability of velocities. The proposed NN estimation model can optimize its structure by adjusting the number of neurons through a self-structure strategy, which is used to estimate unknown nonlinear functions caused by unmodeled dynamics, uncertain model parameters, and external unknown environmental disturbances. Based on the SNN error estimation model, the proposed USV dynamic controller has an a priori bound, which effectively avoids the saturation of the controller. The main result analysis shows that the whole closed-loop error system is ISS. The experimental simulation results verify the effectiveness of the control algorithm. Further work will consider the influence of factors such as noise, communication delay, and actuator failure on the controller.

## Figures and Tables

**Figure 1:** Neuron adjustment schematic diagram.

**Figure 2:** SNN neuron algorithm strategy flowchart.

**Figure 3:** Illustration of USV for target tracking.

**Figure 4:** Control scheme schematic diagram.

**Figure 5:** Formation structure of the leader and follower.

**Figure 6:** USV trajectories.

**Figure 7:** Dynamic estimation of uncertain targets based on ESO.

**Figure 8:** SNN performance of SNN when approximating unknown nonlinear function *F*.

**Figure 9:** Control input.

**Figure 10:** Number of USV neurons.

**Figure 11:** Target-tracking errors.

**Figure 12:** RBFNN performance when approximating unknown nonlinear function *F*.

**Figure 13:** Approximation errors by the SNN and RBFNN.

**Figure 14:** Comparisons of the target-tracking error *z*_*d*_.

**Figure 15:** Comparisons of the target-tracking error *z*_*ψ*_.

**Figure 16:** Comparisons of the control input *τ*_*u*_.

**Figure 17:** Comparisons of the control input *τ*_*r*_.

## Data Availability

The data used to support the findings of this study are included within the article.
